The article "Temperature Changes in Oral All-Ceramic Materials with Different Optical Properties under Er:YAG Laser Irradiation" was published in 2022. Journal: Dis Markers.

# Temperature Changes in Oral All-Ceramic Materials with Different Optical Properties under Er:YAG Laser Irradiation

**DOI:** 10.1155/2022/3443891

**Published:** 2022-09-12

**Authors:** Shuo Yang, Zhaoqiang Yun, Lei Zhao, Mingwei Cheng, Tengfei Zhou, Erliang Huang, Yongtong Guo, Yan Xu, Wuwei Yin, Xiao Chen, Junchen Wang, Hongxing Chu

**Affiliations:** ^1^Center of Oral Implantology, Stomatological Hospital, Southern Medical University, Guangzhou, China; ^2^School of Biomedical Engineering, Southern Medical University, Guangzhou, China; ^3^Department of Periodontics-Implantology, Stomatological Hospital, Southern Medical University, Guangzhou, China; ^4^Guangzhou Women and Children's Medical Center, Guangzhou, China; ^5^The Fourth Affiliated Hospital of Guangzhou Medical University, Guangzhou, China; ^6^School of Mechanical Engineering and Automation, Beihang University, Beijing, China

## Abstract

**Objectives:**

This in vitro study is aimed at assessing the oral all-ceramic materials energy transmission and temperature changes after Er:YAG laser irradiation of monolithic zirconia all-ceramic materials with varying optical properties.

**Materials and Methods:**

Two monolithic zirconia materials, Zenostar T and X-CERA TT (monolithic Zirconia), were studied. Specimens were divided into four groups, with a thickness of 1.0, 1.5, 2.0, and 2.5 mm, respectively. The chemical elemental composition of the two materials was determined using X-ray spectroscopy and Fourier transform infrared spectroscopy. The light transmittance of specimens with different thicknesses was measured using a spectrophotometer at three wavelength ranges: 200–380, 380–780, and 780–2500 nm. Irradiation with Er:YAG laser was performed, and the resultant temperature changes were measured using a thermocouple thermometer.

**Results:**

Compositional analysis indicated that Si content in X-CERA TT was higher than that in Zenostar T. The light transmittance of both materials decreased as specimen thickness increased. Er:YAG laser irradiation led to temperature increase at both Zenostar T (26.4°C–81.7°C) and X-CERA TT (23.9°C–53.5°C) specimens. Both optical transmittance and temperature changes after Er:YAG laser irradiation were consistent with exponential distribution against different thickness levels.

**Conclusion:**

Er:YAG laser penetration energy and resultant temperature changes were mainly determined by the thickness and composition of the examined monolithic zirconia materials.

## 1. Introduction

Dental ceramic materials exhibit excellent aesthetics and biocompatibility [1]. Rapid advances in material science technology and reduction in prices have facilitated the widespread use of all-ceramic materials in various clinical settings within restorative dentistry. The utilization of all-ceramic materials in restorative dentistry is highly prevalent and a chief modality in clinical restorative practice owing to excellent material properties and clinical performance. Multiple studies have indicated good long-term clinical success and found 5-year failure rates of all-ceramic restorations are around 9% [2–5], primarily occurring due to porcelain splitting and prosthesis debonding. These complications often necessitate the removal of all-ceramic restorations [6, 7]. In addition, other complications can also necessitate restoration removal. A very common complication is secondary caries at the crown margins. At present, the main method of dismantling the prosthesis is violent disassembly, during which a great number of vibrations occur, and this is uncomfortable for patients. Additionally, the disassembly process is time-consuming and labour intensive. Importantly, if improperly performed, the underlying tooth structure might be damaged during this procedure.

The article "Temperature Changes in Oral All-Ceramic Materials with Different Optical Properties under Er:YAG Laser Irradiation" was published in 2022. Journal: Dis Markers.

Lasers have attained widespread application in dentistry in recent decades [8, 9]. Lasers have been found safe for the ablation of dental hard tissue and composite resins when used in the right mode [10, 11]. In vitro experiments have displayed that laser removal of all-ceramic restorations is feasible [12–14]. This is attributable to the fact that all-ceramic materials possess varying degrees of transparency. Laser energy can partially transmit through an all-ceramic restoration body to ablate the underlying adhesive, which can enable easy separation of the all-ceramic abutment [15] (Figure 1). Clinically, Morford et al. have demonstrated the application of Er:YAG laser to remove all-ceramic veneers with excellent results [16]. Similarly, Cranska has shown that laser application could facilitate rapid and easy removal of all-ceramic crowns [17]. Others have shown that laser application enabled the rapid removal of orthodontic all-ceramic brackets and postulated the mechanistic basis of adhesive material heat ablation occurring under laser irradiation [18]. These studies indicate that as compared with the conventional method, the use of lasers can enable the removal of all ceramic restorations in a shorter timespan with greater efficiency and lower risk of damage to the abutment tooth structure or the surrounding soft and hard tissues. Considering these advantages, rapid growth in the application of dental lasers for managing complications involving all-ceramic restorations can be anticipated.

At the same time, the laser removal process induces transient occurrence of high temperatures, which can injure surrounding soft and hard tissues, particularly if improper laser energy settings are used resulting in a very high temperature change. In general, tissue denaturation occurs within seconds if biological tissue temperature exceeds 60°C, and such change is irreversible. Several researchers have addressed this issue. Previous work [19] has explored the effects of an instantaneous increase in temperature on the teeth and pulp during laser removal of all-ceramic restorations. Others have shown that dental pulp tissue maintained its biological activity if the temperature rise was lower than 5.6°C [20]. When the temperature rise exceeded 16°C, all pulp tissue activity was lost. The temperature rise in the pulp cavity could be controlled at approximately 5.6°C when all-ceramic restorations were removed by using appropriate Er:YAG laser energy [21]. In our previous study, we found that Er:YAG laser could remove all-ceramic restorations but led to transient high temperatures locally [22]. If laser power is excessively high or irradiating time is excessively long, along with the remaining adhesive, underlying tooth structure may be carbonized, and tissues including enamel, dentin, or pulp can be subject to irreversible damage, leading to complications. Thus, a detailed understanding of laser parameters and their effects on temperature rise in different ceramic materials is essential to apply laser-assisted restoration removal.

The article "Temperature Changes in Oral All-Ceramic Materials with Different Optical Properties under Er:YAG Laser Irradiation" was published in 2022. Journal: Dis Markers.

Among various all-ceramic materials, monolithic zirconia has gained widespread popularity owing to its high flexural strength, superior esthetics, and monolithic properties, which avoid chipping [23]. Of note, varying clinical conditions and aesthetic requirements demand differing esthetic requirements, based on which monolithic zirconia materials with varying optical properties might be selected. Our previous experiments have confirmed that Er:YAG laser can remove all-ceramic restorations effectively but the transmission of heat through the material can adversely affect the adjacent and underlying tissues. However, whether and how monolithic zirconia materials with different optical properties vary in laser energy penetrated when Er:YAG laser is applied for restoration removal is not understood. Therefore, the present study was designed to evaluate temperature changes at monolithic zirconia all-ceramic materials with different optical properties under Er:YAG laser irradiation and thus provide preliminary evidence and guidance for clinical settings.

## 2. Materials and Methods

The two kinds of monolithic zirconia all-ceramic materials with different optical properties were used in this experiment. These included Zenostar T (Ivoclar Vivadent, Switzerland) and X-CERA TT (Xtcera, China). 10 mm × 10 mm blocks with a thickness of 1.0, 1.5, 2.0, or 2.5 mm were prepared using a CAD/CAM system. Three samples were prepared for each thickness, resulting in a total of 24 blocks. The sample's thickness was measured with a vernier calliper, and measurement error was controlled within ±0.02 mm. After preparation, the samples were placed in distilled water, ultrasonically cleaned for 10 minutes, and air-dried. The samples were processed at the Technical Center of Stomatological Hospital, Southern Medical University.

The article "Temperature Changes in Oral All-Ceramic Materials with Different Optical Properties under Er:YAG Laser Irradiation" was published in 2022. Journal: Dis Markers.

Determination of physical and chemical characteristics: the chemical composition of the samples was determined by X-ray spectroscopy and Fourier transformed infrared (FTIR) spectroscopy. The elemental composition, proportion, and chemical composition were analyzed. The surface morphology was observed using scanning electron microscopy (SEM).

Optical performance test: a spectrophotometer (LAMBDA 750, PerkinElmer, USA) was used in the ultraviolet (200–380 nm), visible (380–780 nm), and infrared regions (780–2500 nm). Blocks of each material type and thickness were examined at the three different wavelengths to obtain the light transmittance. Each block was measured thrice at the same wavelengths and averaged.

Temperature measurement: the wavelength of the Er:YAG laser (Fidelis Plus III, Fotona, Slovenia) used was 2940 nm, with the frequency set to 15 Hz, and the pulse width at 330 *μ*s. A laser handpiece was utilized to control the diameter of the laser spot at 1 mm. The laser was placed at 7 mm directly above the sample and irradiated perpendicular to the sample's surface. Each sample was irradiated thrice at different locations under the conditions of no water/gas cooling. The duration of one irradiation was 5 s. The laser energy was progressively increased from 50 mJ to 250 mJ at increments of 50 mJ. A thermometer probe was attached to the back of the sample, and a thermocouple thermometer was used to measure the temperature changes after the laser penetrated the samples. All laser-specific safety measures were observed during the procedure. All temperature measurements were performed at room temperature.

The FTIR and light transmittance test equipment were provided by the Central Laboratory of the Southern Medical University of Technology. Data analysis was performed using SPSS17.0.

## 3. Results

### 3.1. Physical and Chemical Characteristics

X-ray energy spectrum analysis: Table 1 shows the results of X-ray spectrum analysis. Zr and O were the main chemical elements for both materials. The main components of Zenostar T were Zr and O, accounting for 46.2% and 32%, respectively. The minor elements consisted of C (19.8%), Si (1.3%), and small amounts of other elements. X-CERA TT contained Zr (44.7%) and O (30.2%) and C (15.6%). Compared with Zenostar T, X-CERA TT contained more Si (8.6%). X-ray energy spectrum analysis showed that the elemental composition of Zenostar T and X-CERA TT samples were similar, with the main components being Zr oxide.

The article "Temperature Changes in Oral All-Ceramic Materials with Different Optical Properties under Er:YAG Laser Irradiation" was published in 2022. Journal: Dis Markers.

#### 3.1.1. FTIR

Figure 2 shows the FTIR spectra of Zenostar T and X-CERA TT samples. Both Zenostar T and X-CERA TT samples showed a characteristic peak of Zr dioxide at 600–605 nm, which was ascribed to the Zr–O stretching, indicating that both samples were materials constituted mainly of Zr dioxide. Both Zenostar T and X-CERA TT samples displayed a longer range of strong peaks at 1258–1537 nm, revealing the carbonate structure. The FTIR results revealed that both the structural component and the chemical group were nearly the same, except that X-CERA TT samples exhibited a peak elevation at 3500–3750 nm, which was attributed to the stretching of the Si–OH group vibration. This finding indicated that typical silicon-containing groups were found in X-CERA TT samples. In conjunction with the X-ray spectroscopy results, this finding confirmed that X-CERA TT contained more Si than Zenostar T.

#### 3.1.2. SEM

Figures 3(a) and 3(b) show the SEM images for Zenostar T and X-CERA TT at 1000-fold magnification. The surface morphology of Zenostar T was smoother and contained a small amount of highlighted particles. X-CERA TT presented numerous highlighted particles, which were small in size, randomly distributed throughout the material's surface, and displayed a grainier appearance. The surface morphologies of both materials remained undamaged after laser irradiation.

#### 3.1.3. Light Transmittance Test

Standard light sources of different wavelengths, namely, ultraviolet (200–380 nm), visible light (380–760 nm), and infrared (760–2500 nm), were used in the test and assessed. The light transmittance of Zenostar T and X-CERA TT samples was detected with a spectrophotometer (Lambda 750, PerkinElmer, USA).

The ultraviolet transmittance of Zenostar T and X-CERA TT samples was found inversely proportional to the sample thickness. A high thickness corresponded to a low ultraviolet transmittance. The ultraviolet transmittance of Zenostar T was close to that of X-CERA TT (between 0.5% and 1.4%). In some cases, the transmittance of the two samples was similar at the same thickness. In general, the transmittance of Zenostar T samples was slightly higher than that of X-CERA TT under ultraviolet irradiation.

The visible light transmittance of the X-CERA TT and Zenostar T samples ranged from 0.9% to 1.6% and 0.9% to 1.3%, respectively, and X-CERA TT showed higher values than Zenostar T. For both materials, the visible light transmittance decreased as the thickness of the samples increased.

The article "Temperature Changes in Oral All-Ceramic Materials with Different Optical Properties under Er:YAG Laser Irradiation" was published in 2022. Journal: Dis Markers.

The infrared transmittance of the X-CERA TT samples was significantly higher than that of Zenostar T. Specifically, at a 1 mm sample thickness, the infrared transmittance of X-CERA TT samples was 5.1%, while that of the Zenostar T samples was 1.8%. However, as sample thickness increased, the infrared transmittance of the X-CERA TT samples declined more rapidly. In general, the infrared transmittance of both types of samples decreased with increasing thickness.

Figure 4 shows the exponential fitting results for the light transmittance irradiated by ultraviolet light (200–380 nm, Figure 4(a)), visible light (380–760 nm, Figure 4(b)), and infrared light (760–2500 nm, Figure 4(c)) for the Zenostar T and X-CERA TT samples. The goodness-of-fit of all fitting curves, r2, exceeded 0.95, which indicated high goodness of fit range. Such a good fit implied that the light transmittance of Zenostar T and X-CERA TT samples was consistent with exponential distribution at different thicknesses.

As thickness increased, the integral light transmittance of samples declined under all types of light irradiation. Under the irradiation wavelength of 200–380 nm, the light transmittance of Zenostar T was higher than that of X-CERA TT. As the light wavelength increased, the light transmittance of X-CERA TT samples gradually increased and remained higher than that of Zenostar T.

#### 3.1.4. Temperature Changes during Laser Irradiation

In this experiment, the laser energy was initially set to 50 mJ and progressively increased to 250 mJ at increments of 50 mJ. The laser source was placed at a distance of 7 mm perpendicularly above the samples, and the surface was irradiated for 5 s without water/gas physical cooling. Each sample was irradiated thrice at different locations on its surface. The temperature change during irradiation was recorded by a thermocouple thermometer. The starting temperature (ambient temperature) of the thermocouple probe was 18.6°C. At the start of each measurement, the temperature of the thermocouple probe was returned to the initial temperature.

The temperature at Zenostar T samples ranged from 26.4°C to 81.7°C for the thickness range of 1–2.5 mm under the irradiation energy of 50–250 mJ. The temperature range at X-CERA TT samples was 23.9°C–53.5°C under the same conditions. Greater sample thickness corresponded to smaller temperature change. Under the same laser energy, Zenostar T samples exhibited a greater temperature change than X-CERA TT.

The article "Temperature Changes in Oral All-Ceramic Materials with Different Optical Properties under Er:YAG Laser Irradiation" was published in 2022. Journal: Dis Markers.

For samples of the same thickness, the recorded temperature increased as the laser irradiation energy increased. For Zenostar T samples at 1 mm, the difference in recorded temperatures was 49.8°C under the irradiation energies of 250 and 50 mJ. However, the difference in recorded temperatures was 23.8°C for X-CERA TT samples under the same condition. Differences in the temperature changes were 13.3°C and 11.2°C, respectively, for Zenostar T and X-CERA TT samples under the irradiation energies of 250 and 50 mJ at 2.5 mm thickness. When Er:YAG laser with a 50 mJ energy was used for irradiation of 1 and 2.5 mm thick samples, the temperature measurements were 33.43°C + 1.30°C (mean ± SD) and 26.88°C + 1.32°C (mean ± SD) for Zenostar T and 28.7°C + 0.50°C (mean ± SD) and 23.9°C + 1.02°C (mean ± SD) for X-CERA TT.

Figure 5 shows the exponential fitting curve of the temperature changes of Zenostar T and X-CERA TT samples for different thicknesses under different laser irradiation energies. Er:YAG laser irradiation of the Zenostar T(Figure 5(a)) and X-CERA TT (Figure 5(b)) samples led to a temperature increase that was inversely proportional to the sample thickness and directly proportional to laser power.

## 4. Discussion

The present study demonstrated that Er:YAG laser penetration energy and its resulting temperature changes were dependent upon the thickness and composition of the examined monolithic zirconia materials. These findings offer important directions for clinical applications to avoid iatrogenic injury to tissues during restoration removal with Er:YAG lasers. To our knowledge, this study is the first to evaluate temperature changes at all-ceramic materials with different optical properties under Er:YAG laser irradiation.

Using X-ray spectrum elemental detection, we demonstrated that the elemental composition of Zenostar T and X-CERA TT were similar, comprising Zr, O, C, Si, and other elements. Furthermore, FTIR spectroscopy showed that both Zenostar T and X-CERA TT samples contained large amounts of Zr oxide groups. Physical and chemical analyses confirmed that Zr oxide was the main component of both Zenostar T and X-CERA TT. Of note, X-CERA TT samples contained a higher amount of Si, which was approximately 6–7 times that in Zenostar T. This was also demonstrated by the FTIR spectra, where as compared to Zenostar T, X-CERA TT manifested a rising peak resulting from the stretching vibration of the Si-containing groups at 3500–3750 nm. These differences in composition would account for differences in optical properties, and thus might affect material selection in different clinical situations. Electron microscopy analysis showed that the surface of Zenostar T was uniform with a few scattered particles of different sizes, whereas the surface of X-CERA TT displayed numerous bright particles that were more evenly distributed, smaller, and more uniform than those of Zenostar T. These differences could arise from the differences in material composition. In a related finding, Stoia et al. [24] showed that the presence of Si inhibited the agglomeration of ZrO_2_ particles, and the size of the ZrO_2_ particles modified by SiO_2_ was smaller than that of unmodified ones. In alignment, X-ray spectroscopy, FTIR, and electron microscopy data confirmed that X-CERA TT contained more Si than Zenostar T, and the former presented a more even surface with smaller particles.

The article "Temperature Changes in Oral All-Ceramic Materials with Different Optical Properties under Er:YAG Laser Irradiation" was published in 2022. Journal: Dis Markers.

All-ceramic materials can achieve good restorative aesthetics because of their high relative transparency. Light comprises electromagnetic waves consisting of different wavelengths including infrared, visible light, and ultraviolet light. The transparency of all-ceramic materials allows light to partially reflect, absorb, and transmit. All-ceramic materials' chemical characteristics, crystal number and diameter, porosity, and sintering density determine the optical properties of light reflection, absorption, scattering, and transmission rate [23]. By adjusting trace elements or the crystal phase, all-ceramic materials can be designed to manifest different optical properties. The light transmittance of materials can be determined by a spectrometer from the measurement of spectral power transmission or reflectance. In this study, we found that the amount of Si in Zenostar T was significantly lower than that in X-CERA TT. Si is a good infrared optical material. Previous studies have highlighted that the infrared transmittance of ultrapure silicon can reach as high as 90%–95% and that the UV transmittance in silica does not exceed 30% [25, 26]. Zenostar T had a relatively high transmittance under ultraviolet irradiation. However, under infrared irradiation, the transmittance of the X-CERA TT samples was significantly higher than that of Zenostar T, which is attributable to the difference in composition and crystalline phase. Lambert's law states that at a certain wavelength, the amount of light absorbed is proportional to the material thickness [27]. Light transmittance is closely related to material characteristics and sample thickness [28, 29]. Here, sample thickness was found exponentially related to the transmittance, and as sample thickness increased, the transmittance decreased for both materials under all types of light sources. The light transmission rates for both Zenostar T and X-CERA TT samples increased exponentially with sample thicknesses, indicating that optical properties were determined by material thickness.

The article "Temperature Changes in Oral All-Ceramic Materials with Different Optical Properties under Er:YAG Laser Irradiation" was published in 2022. Journal: Dis Markers.

Possessing a wavelength of 2.94 *μ*m within the infrared range, Er:YAG laser has wide applications in dental practice [30, 31]. One emerging clinical application comprises the removal of all-ceramic restorations. In this experiment, the Er:YAG laser frequency was set at 15 Hz, and the pulse width was 330 *μ*s. The laser spot diameter was controlled at 1 mm by a laser handpiece. The energy was set to 50 mJ and progressively increased to 250 mJ. These parameters were carefully selected to simulate routine clinical settings. Of note, the temperature change was measured by a thermocouple thermometer, which had high sensitivity and accuracy, and has been widely used in similar experiments. Therefore, the results can be considered a good representative of temperature changes occurring in clinical situations.

Comparative analysis of the measured temperature at the Zenostar T and X-CERA TT samples for different thicknesses showed that under the same Er:YAG laser irradiation energy and for the sample thickness range of 1–2.5 mm, the amplitude of temperature increase at Zenostar T was higher than that at X-CERA TT. The maximum temperature difference between the two kinds of materials was 30.5°C, which occurred at a thickness of 1 mm under the highest applied irradiation energy of 250 mJ. The minimum temperature difference between the two materials was 2.2°C, occurring at a sample thickness of 2.5 mm under the irradiation energy of 50 mJ. As sample thickness decreased and laser irradiation energy increased, the measured temperature at Zenostar T sample displayed a higher growth rate than that at X-CERA TT. This difference may be attributed to the earlier described differences in the chemical and physical properties of the two materials. The major component of both Zenostar T and X-CERA TT was Zr oxide, while X-CERA TT contained more Si. Zr is a metal element with a specific heat of 0.27 J/gK and thermal conductivity of 0.227 W/cmK. Si is a nonmetallic element with a specific heat of 0.71 J/gK and thermal conductivity of 1.48 W/cmK. The heat transmission of Zr and its oxide is better than that of Si, which would account for the greater rise in temperature, as Zenostar T had a higher Zr amount, and X-CERA TT sample had a higher Si amount. Furthermore, the differences in physical and surface properties may also have contributed to the greater temperature change in Zenostar T leading to higher heat conductance. Comparing Zenostar T and X-CERA TT at the sample thickness range of 1–2.5 mm which are commonly used in dental restorations, we demonstrated that temperature changes induced by Er:YAG laser penetration were associated with the physical and chemical characteristics of monolithic zirconia. These findings provide a preliminary basis for devising clinical protocols for laser-assisted all ceramic restoration removal based on individual material properties, to avoid iatrogenic damage to tissues. Furthermore, Er,Cr:YSGG laser has also been used for the removal of restorations, and future studies should identify its parameters relevant to different materials [32]. Importantly, in earlier work, a laser-induced temperature rise greater than 5.5°C was shown to cause injury to pulpal tissue [21] but such temperatures were noted only when the water jet was misdirected, so the authors suggested the use of cooled water. The temperature rises noted in the current study were higher than this threshold, highlighting the need for a detailed understanding of effects of restorative material property and thickness on pulpal temperature change. These findings also highlight the necessity of developing stringent clinical protocols for laser-assisted restoration removal with adequate cooling, which take into account specific material characteristics.

The article "Temperature Changes in Oral All-Ceramic Materials with Different Optical Properties under Er:YAG Laser Irradiation" was published in 2022. Journal: Dis Markers.

The present work was limited to two monolithic zirconia material types with varying optical, physical, and chemical properties and a single laser. In practice, an increasingly large number of all ceramic material types are available. Future studies should characterize the laser penetration energy at a larger variety of such materials to expand knowledge of the parameters that can influence the success laser-assisted restoration removal. Furthermore, the present study is an in vitro experiment with very controlled conditions. In clinical situations, a number of other variables may come into play. Clinical studies are essential to develop safe and effective laser-assisted restoration removal protocols.

## 5. Conclusion

All-ceramic restorations at the thickness range of 1.0–2.5 mm are widely used in clinical practice. Under 50–250 mJ Er:YAG laser irradiation for 5 s, the temperature of Zenostar T and X-CERA TT samples increased to 26.4°C–81.7°C and 23.9°C–53.5°C, respectively. Oral tissues can be subject to iatrogenic injury in the absence of effective cooling under these conditions. No obvious correlation was found between Er:YAG laser penetration energy and the optical properties of the materials. Furthermore, the optical properties of the materials did not significantly influence laser energy in simulated clinic settings. The penetration energy of Er:YAG laser was mainly determined by the physical and chemical characteristics of the materials. These findings underscore a need to take material properties into account in the development of clinical protocols for laser-assisted restoration removal.

The article "Temperature Changes in Oral All-Ceramic Materials with Different Optical Properties under Er:YAG Laser Irradiation" was published in 2022. Journal: Dis Markers.

## Figures and Tables

**Figure 1:** Clinical case showing laser removal of all-ceramic restorations.

**Figure 2:** The FTIR spectra of Zenostar T and X-CERA TT.

**Figure 3:** SEM images of Zenostar T (a) and X-CERA TT (b) ×1000.

**Figure 4:** Exponential distribution of light transmittance for Zenostar T and X-CERA TT samples. Ultraviolet transmittance (a). Visible light transmittance (b) and infrared transmittance (c).

**Figure 5:** Exponential distribution of temperature changes at Zenostar T (a) and X-CERA TT (b) samples.

**Table 1:** Chemical element compositions of Zenostar T and X-CERA TT.

Material	Average mole percentage (%)				
	Zr	O	C	Si	Others
Zenostar T	46.2	32	19.8	1.3	0.7
X-CERA TT	44.7	30.2	15.6	8.6	0.9

## Data Availability

The data that support the findings of this study are available from the corresponding author (H Chu), upon reasonable request.
